The article "Evaluation of the Replication, Pathogenicity, and Immunogenicity of Avian Paramyxovirus (APMV) Serotypes 2, 3, 4, 5, 7, and 9 in Rhesus Macaques" was retracted in 2020. Reasons: manipulated images; duplicated images; concerns about the data.

# Evaluation of the Replication, Pathogenicity, and Immunogenicity of Avian Paramyxovirus (APMV) Serotypes 2, 3, 4, 5, 7, and 9 in Rhesus Macaques

**DOI:** 10.1371/journal.pone.0075456

**Published:** 2013-10-10

**Authors:** Sunil K. Khattar, Baibaswata Nayak, Shin-Hee Kim, Sa Xiao, Sweety Samal, Anandan Paldurai, Ursula J. Buchholz, Peter L. Collins, Siba K. Samal

**Affiliations:** 1 Virginia-Maryland Regional College of Veterinary Medicine, University of Maryland, College Park, Maryland, United States of America; 2 Laboratory of Infectious Diseases, National Institute of Allergy and Infectious Diseases, Bethesda, Maryland, United States of America; Thomas Jefferson University, United States of America

## Abstract

Avian paramyxoviruses (APMV) serotypes 1–9 are frequently isolated from domestic and wild birds worldwide. APMV-1 (also called Newcastle disease virus, NDV) is attenuated in non-human primates and is being developed as a candidate human vaccine vector. The vector potential of the other serotypes was unknown. In the present study, we evaluated nine different biologically- or recombinantly-derived APMV strains for the ability to replicate and cause disease in rhesus macaque model. Five of the viruses were: biologically-derived wild type (wt) APMV-2, -3, -5, -7 and -9. Another virus was a recombinant (r) version of wt APMV-4. The remaining three viruses were versions of wt rAPMV-2, -4 and -7 in which the F cleavage site had been modified to be multi-basic. Rhesus macaques were inoculated intranasally and intratracheally and monitored for clinical disease, virus shedding from the upper and lower respiratory tract, and seroconversion. Virus shedding was not detected for wt APMV-5. Very limited shedding was detected for wt rAPMV-4 and modified rAPMV-4, and only in a subset of animals. Shedding by the other viruses was detected in every infected animal, and usually from both the upper and lower respiratory tract. In particular, shedding over a number of days in every animal was observed for modified rAPMV-2, wt APMV-7, and modified rAPMV-7. Modification of the F protein cleavage site appeared to increase shedding by wt rAPMV-2 and marginally by wt rAPMV-4. All APMVs except wt APMV-5 induced a virus-specific serum antibody response in all infected animals. None of the animals exhibited any clinical disease signs. These results indicate that APMVs 2, 3, 4, 7, and 9 are competent to infect non-human primates, but are moderately-to-highly restricted, depending on the serotype. This suggests that they are not likely to significantly infect primates in nature, and represent promising attenuated candidates for vector development.

## Introduction

The avian paramyxoviruses (APMVs) are isolated from wild and domestic birds all over the world. The APMVs have been divided into nine serotypes (APMV 1 to 9) based on hemagglutination inhibition (HI) and neuraminidase inhibition (NI) assays [1]. More recently, viruses representing potential APMV serotypes 10 and 11 were isolated from Rockhopper Penguins [2] and common teal [3], respectively. APMV-1, which includes all strains of Newcastle disease virus (NDV), has been extensively characterized because virulent NDV strains cause severe disease in chickens. NDV strains are divided into three pathotypes based on their virulence in chickens: highly virulent (velogenic) strains cause severe respiratory and neurologic diseases; moderately virulent (mesogenic) strains cause milder disease, and nonpathogenic (lentogenic) strains cause inapparent infection. Mesogenic and lentogenic strains of NDV are highly restricted for replication and highly attenuated in non-avian species including primates, and are being developed as vaccine vectors for animal and human pathogens. Previous studies have shown that APMV serotypes 2-9 replicate not only in avian species, but also in mice and hamsters [4], [5]. However, their ability to replicate and possibly cause disease in primates, and their potential as human vaccine vectors, were unknown.

The article "Evaluation of the Replication, Pathogenicity, and Immunogenicity of Avian Paramyxovirus (APMV) Serotypes 2, 3, 4, 5, 7, and 9 in Rhesus Macaques" was retracted in 2020. Reasons: manipulated images; duplicated images; concerns about the data.

The APMVs belong to family *Paramyxoviridae*, a large and diverse family that includes viruses from a wide variety of mammalian, avian, reptilian, and fish species around the world [6]. Some members of the family are responsible for major human and animal diseases, while others cause inapparent infections. Paramyxoviruses are pleomorphic and enveloped and contain a non-segmented, negative-sense, single-stranded RNA genome of 13–19 kb. On the basis of virus structure, genome organization and sequence relatedness, the family *Paramyxoviridae* is divided in to two subfamilies: *Paramyxovirinae and Pneumovirinae* [6]. The subfamily *Paramyxovirinae* is divided into five genera: *Respirovirus* (including Sendai virus and human parainfluenza virus types 1 and 3), *Rubulavirus* (including parainfluenza virus 5 [previously known as simian virus type 5], mumps virus, and human parainfluenza virus types 2 and 4), *Morbillivirus* (including measles and canine distemper viruses), *Henipavirus* (comprising Hendra and Nipah viruses), and *Avulavirus* (comprising the APMVs). Subfamily *Pneumovirinae* contains two genera, *Pneumovirus* (including human and bovine respiratory syncytial viruses) and *Metapneumovirus* (comprising human metapneumovirus and the avian metapneumoviruses) [6], [7]

Although a lot of information is available for APMV-1, much less is known about the molecular biology, pathogenicity and host range of the other APMV serotypes. As an initial step towards their characterization, we have recently determined the complete genome sequences of APMV-2 to -9 [8]–[15] and we have developed reverse genetics systems for APMV-2, -3, -4 and -7 [16]–[19]. However, the biological characteristics and pathogenicity of APMV-2 to -9 remain poorly understood. APMV-2 has been associated with severe respiratory disease, reduced egg production and infertility in turkeys [20], [21]. APMV-3 has been associated with encephalitis and high mortality in caged birds, respiratory disease in turkeys and stunted growth in young chickens [22], [23]. APMV-4 strains have been isolated from chickens, ducks and geese [19]. APMV-5 causes disease in budgerigars that is characterized by depression, dyspnoea, diarrhea and high mortality [24]. APMV-6 and -7 cause mild respiratory disease in turkeys and are associated with a drop in egg production [25], [26]. APMV-8 and -9, isolated from ducks, waterfowl, and other wild birds, did not produce any clinical signs of viral infection in chickens [27], [28]

In the last 10 years, reverse genetic techniques have made it possible to engineer NDV as a potential vaccine vector for both human and animal uses [29]–[39]. NDV vectors expressing a number of foreign antigens have been evaluated not only in avian hosts, but also in murine and nonhuman primate models [29]–[33], [40]–[42]. Several strains of NDV have been shown to be highly restricted for replication in these mammalian models, indicating that they are highly attenuated due to a strong host range restriction and represent promising vaccine vectors. However, NDV strains are highly related antigenically, and therefore the use of NDV vectors for multiple purposes would be compromised by the induction of vector-specific immunity. This limitation might be overcome by using other APMV serotypes that are antigenically distinct from NDV as alternative vaccine vectors. In addition, it is possible that one or more of the other APMV serotypes might have other advantageous properties that cannot be predicted, such as increased immunogenicity compared to NDV. Furthermore, the possibility exists that one or more of the other APMV serotypes might be pathogenic in certain non-avian hosts including primates. For example, an APMV-2-like virus was previously recovered from a cynomolgus monkey with respiratory disease [43], and an APMV-3-like virus was recovered from pigs [44]. Therefore, evaluation of APMV-2 to -9 in non-avian species was warranted.

The article "Evaluation of the Replication, Pathogenicity, and Immunogenicity of Avian Paramyxovirus (APMV) Serotypes 2, 3, 4, 5, 7, and 9 in Rhesus Macaques" was retracted in 2020. Reasons: manipulated images; duplicated images; concerns about the data.

We recently showed that APMV-2 to -9 are competent to infect and replicate to low-to-moderate titers in mice and hamsters [37], [38]. However, rodents are uncertain predictors of performance in other species such as humans because it is possible, and indeed likely, that there will be differences in the level of host range restriction between rodents and other species including primates. In the present study, we sought to evaluate the replication and pathogenicity of APMV-2, -3, -4, -5, -7 and -9 in rhesus macaques as a surrogate for humans. The viruses included biologically- and recombinantly-derived wt viruses as well as several recombinant viruses in which the F protein cleavage site had been modified to be multi-basic and to contain the optimal furin protease cleavage site motif RX(R/K)R↓ (signature R and K residues underlined). This was done because the presence of a furin motif in the F protein cleavage site typically facilitates cleavage and is a major determinant of virulence for NDV strains [45], [46], although this paradigm is uncertain for the other APMV serotypes [16], [18], [19]. The present study showed that, except for APMV-5, all of the APMVs under evaluation replicated at varying levels in rhesus macaques without inducing any apparent clinical disease signs. Thus, APMV serotypes 2, 3, 4, 7, and 9 are infectious, replication-competent and attenuated in non-human primates. In future work, the reverse genetics system for APMV-2, -4, and -7 will be used for the development of APMV vectored vaccines.

## Materials and Methods

### Ethical Statement

Adult rhesus macaques (Macaca mullatta) were obtained from the NIAID breeding colony located on Morgan Island, SC. This colony is AAALAC international accredited and OLAW assured. All animals are transported in accordance with USDA guidelines and permits. The non-human primate experiments were performed at a site approved by the Association for Assessment and Accreditation of Laboratory Animal Care International, with a protocol approved by the Animal Care and Use Committee of the National Institute of Allergy and Infectious Diseases. Since this study involved infectious agents, rhesus macaques were housed individually in microisolator cages for the duration of the study. This was necessary to prevent transmission of respiratory viruses to other non-human primates in the room and to animal handlers. All monkeys were able see other monkeys of the same species. Monkeys were on an environmental enrichment program (additional objects for manipulation, perches, food enrichment). Animals were observed at least two times a day by animal care staff for any illnesses or abnormalities. No animals were sacrificed for this study.

All the experiments where 9-day old embryonated chicken eggs were used ended on or before day 13. Before collecting allantoic fluid from the eggs, the embryos were sacrificed by incubating the eggs at 4°C in a refrigerator for 2 hour.

The article "Evaluation of the Replication, Pathogenicity, and Immunogenicity of Avian Paramyxovirus (APMV) Serotypes 2, 3, 4, 5, 7, and 9 in Rhesus Macaques" was retracted in 2020. Reasons: manipulated images; duplicated images; concerns about the data.

### Cells and viruses

Chicken embryo fibroblast (DF-1) and African green monkey kidney (Vero) cell lines, obtained from the American Type Culture Collection (ATCC, Manassas, VA), were grown in Dulbecco's modified Eagle medium (DMEM) containing 10% fetal bovine serum (FBS) and maintained in DMEM with 5% FBS.

Nine APMV strains were used in this study (see Table 1), all of which had been constructed in previous work: (i) biologically-derived wt APMV-2 strain chicken/Yucaipa/California/56 [8]; (ii) a recombinant derivative of wt APMV-2, called rAPMV-2 (type 1 Africa), in which the natural cleavage site was replaced by the cleavage site RRRRR↓F that is present in a APMV type 1 strain isolated in Africa [16]; (iii) biologically-derived wt APMV-3 strain parakeet/Netherland/449/75 [9]; (iv) recombinant wt APMV-4 strain duck/Hong Kong/D3/75 [10]; (v) a derivative of rAPMV-4, called rAPMV-4/Fc-BC, in which its natural cleavage site was replaced by the cleavage site RRQKR↓F that is present in mesogenic NDV strain Baudette C [19]; (vi) biologically-derived wt APMV-5 strain budgerigar/Kunitachi/74 [11]; (vii) biologically-derived wt APMV-7 strain dove/Tennessee/4/75 [13]; (viii) a recombinant derivative of wt APMV-7, called rAPMV-7/Fcs-5B in which its natural cleavage site was replaced by the cleavage site RRKKR↓FI present in a velogenic NDV strain Nigeria/95, and which includes an amino acid substitution in the +2 position relative to the cleavage site [18]; and (ix) biologically-derived wt APMV-9 strain duck/New York/22/78 [15]. All the APMV serotypes except serotype 5 were grown in the allantoic cavity of 9-day-old specific-pathogen-free (SPF) embryonated chicken eggs. APMV-5 was grown in Vero cells. The allantoic fluids from infected eggs were collected 72 h post-inoculation and virus titers were determined by hemagglutination (HA) assay. Further, the titers of APMVs were determined by plaque assay on DF-1 cells for APMV-2, -3, -4 and -9 and on Vero cells for APMV-5 and -7. The samples were inoculated in triplicate onto 24-well plates of DF-1 or Vero cells at 80% confluency and virus titer was determined by either plaque assay or immunostaining with N specific antibodies.

**Table 1:** APMV strains, F protein cleavage sites, and protease dependence.

APMV strain	F protein cleavage site†	Furin motif	Exogenous protease required *in vitro*
APMV-2	DKPASR FVG	No	No
rAPMV-2 (type 1 Africa)*	DRRRRR FVG*	Yes	No
APMV-3	ARPRGR LFG	No	Yes
APMV-4	ADIQPR FIG	No	No
APVM-4/Fc-BC*	ARRQKR FIG*	Yes	No
APMV-5	GKRKKR FVG	Yes	No
APMV-7	TLPSSR FAG	No	No
APMV-7/Fcs-5B*	TRRKKR FIG*	Yes	No
APMV-9	RIREGR IFG	No	Yes

* The F protein cleavage site was modified to contain the preferred furin motif. Amino acid substitutions are underlined.

† The gap between amino acids in F protein cleavage site indicates position of cleavage.

The article "Evaluation of the Replication, Pathogenicity, and Immunogenicity of Avian Paramyxovirus (APMV) Serotypes 2, 3, 4, 5, 7, and 9 in Rhesus Macaques" was retracted in 2020. Reasons: manipulated images; duplicated images; concerns about the data.

### Infection of rhesus macaques

Adult rhesus macaques (Macaca mulatta) were obtained from Morgan Island. The animals were confirmed to be seronegative for APMV serotypes by hemagglutination inhibition (HI) and plaque reduction assays. The rhesus macaques (4 animals per virus) were infected by the combined intranasal and intratracheal routes using a 1 ml inoculum per site containing 10^6.0^ PFU per mL of the indicated virus, as described previously [47]. Nasal washes (6 ml/animal) and fecal swabs (4 ml/animal) were collected daily on days 0–10, 12, and 21 in phosphate buffered saline (PBS). Bronchoalveolar lavages (BAL; 10 ml/animal) were collected on days 2, 4, 6 and 8 in PBS. Tracheal lavages (3 ml/animal) were collected on days 10, 12 and 21 in PBS. All samples were snap-frozen on dry ice and stored at -80° C until analyzed. Serum samples were obtained on days 0, 21 and 28. Clinical observations were performed daily for 28 days after the inoculation.

### Virus detection and quantification

The nasal wash, BAL, tracheal lavage and fecal samples from each monkey were clarified by centrifugation, and supernatants were collected. The clarified samples were diluted in serial 10-fold dilutions in PBS. The dilutions 10^0^, 10^1^, 10^2^, 10^3^ and 10^4^ (0.1 ml each) were inoculated in triplicate into the allantoic cavity of 9-day-old embryonated chicken eggs. Eggs were incubated at 37°C for 4 days. Allantoic fluid was collected from each egg and the presence of virus was detected by hemagglutination (HA) test with 0.5% chicken RBC. The 50 percent egg infectious dose (EID_50_) virus titer (expressed as log_10_ EID_50_ per mL) was determined by the method of Reed and Muench [48]. Replication of APMV-5 in rhesus monkeys was determined by titration in Vero cells, followed by neuramindase (NA) assay as described by Huang et al., 2004 [49].

### Serological analysis

The serum antibody levels to the specific APMV serotype used for immunization were evaluated pre- and post-immunization by hemagglutination inhibition (HI) assay, virus neutralization (VN) assay, and Western blot analysis, except for the serum antibody response to APMV-5, which was evaluated by VN and by neuraminidase inhibition (NAI) assay. For the HI assay, 25 µl of each serum sample was first treated with 50 µl of receptor destroying enzyme II (catalog number YCC 340–122; Accurate Chemical and Scientific, Westbury NY) at a 1∶3 ratio (vol/vol) at 37°C overnight. Then, 25 µl of 5% sodium citrate was added and incubation was continued at 56°C for 30 min. Each serum sample was allowed to cool to room temperature and 100 µl of packed chicken RBCs were added. After incubation at 4°C for 30 min, samples were centrifuged at 1000 × g for 10 min. Supernatants were used for HI assay. For the HI assay, twofold serial dilutions of treated sera (50 µl) were prepared, and each dilution was combined with 4 HA units of a particular live and homologous APMV serotype. Following 1 h of incubation, 50 µl of 1% chicken RBC was added and incubated for 30 min at room temperature, and HA was scored as the mean reciprocal log_2_ (± standard errors of the mean) of the highest serum dilution causing complete inhibition of four HA units of the indicated APMV.

The article "Evaluation of the Replication, Pathogenicity, and Immunogenicity of Avian Paramyxovirus (APMV) Serotypes 2, 3, 4, 5, 7, and 9 in Rhesus Macaques" was retracted in 2020. Reasons: manipulated images; duplicated images; concerns about the data.

In case of APMV-5, antibody titers were measured by NAI assay. For the NAI assay, APMV-5 strain budgerigar/Kunitachi/74 was used as the source of NA. The NA activity of APMV-5 was measured by a modified fluorometric assay [49]. Briefly, serial twofold dilutions of serum samples were prepared in 20 µl volumes of enzyme buffer (33 mM 2-*N*-morpholino ethanesulfonic acid [MES], pH 6.5, and 4 mM calcium chloride) in a 96-well plate. 20 µl APMV-5, diluted in enzyme buffer to a constant NA amount (an optical density at 450 nm [OD_450_] of 100,000), was added as source of NA, and incubated for 1 h at room temperature. Ten microliters of 12.5% (vol/vol) dimethyl sulfoxide was added to each well of a fluorometric assay plate (black 96-well plates; Microfluor, Franklin, MA). Ten microliters of each serum and virus mixture was transferred in duplicate to the assay plate. 10 µl of diluted virus or enzyme buffer alone were used as positive and negative controls, respectively. The reaction was initiated by the addition of 30 µl of substrate mix [1 volume of 330 mM MES, pH 6.4; 3 volumes of 10 mM calcium chloride; and 2 volumes of 0.5 mM 2′-(4-methylumbelliferyl)-α-d-*N*-acetylneuraminic acid (MUN) (Sigma)] to give a final concentration of 100 µM MUN in the assay. The reaction mixture was incubated at 37°C for 15 min with shaking, and the reaction was terminated by the addition of 150 µl of termination buffer (0.014 M sodium hydroxide in 83% [vol/vol] ethanol). The extent of the reaction was quantified by fluorometry at an excitation wavelength of 360 nm and an emission wavelength of 450 nm using the Victor3 multilabel plate reader (PerkinElmer). Readings from the substrate blanks were subtracted from the virus sample readings. The average background-corrected NA activity was calculated from 12 independent wells. The neuraminidase inhibition (NAI) titer for each sample was reported as the reciprocal log_2_ of the highest serum dilution resulting in a 50% or greater reduction in input NA activity.

The article "Evaluation of the Replication, Pathogenicity, and Immunogenicity of Avian Paramyxovirus (APMV) Serotypes 2, 3, 4, 5, 7, and 9 in Rhesus Macaques" was retracted in 2020. Reasons: manipulated images; duplicated images; concerns about the data.

Neutralizing antibody titers in post-immunization sera collected on day 28 from rhesus macaques were measured in a microneutralization assay. Briefly, 2-fold serial dilutions of 100 µl of heat-inactivated monkey serum samples were mixed with 100 TCID_50_ of the homologous APMV serotype and incubated at 37°C for 1 h. Following incubation, a 50 µl volume of the virus-serum mixture from each serum dilution was added to approximately 150 µl of medium in quadruplicate wells of DF-1 (for APMV-2, -3, -4 and -9) or Vero (for APMV-5 and -7) cells in 96-well plates. The plates were then incubated at 37°C for 72 h and were scored for virus replication based on HA activity of the supernatant. The titer was defined as the the mean reciprocal log_2_ of the highest serum dilution resulting in complete neutralization of infection in 50% of the wells.

Sera from infected rhesus monkeys were further assayed for APMV-specific antibodies by Western blotting. Partially purified APMV (5 µg per lane) were subjected to 10% SDS-PAGE under reducing conditions and transferred to a nitrocellulose membrane. Membrane strips were incubated with a 1∶500 dilution of day 0 and day 28 serum samples from each individual monkey from each group followed by incubation with a 1∶5,000 dilution of HRP-conjugated goat anti-human IgG (Fab specific). The hemagglutinin (HN), fusion (F_0_ and F_1_) nucleocapsid (NP), phophoprotein (P) and matrix (M) proteins specific to a particular APMV serotype were detected by a chemiluminescence assay.

## Results

### Infection of macaques with APMVs and absence of clinical disease

Adult rhesus macaques in groups of four were inoculated by the combined intranasal and intratracheal routes with 10^6^ PFU per site of nine APMV strains representing six serotypes, namely serotypes 2, 3, 4, 5, 7, and 9 (Table 1 and Materials and Methods). Five strains were biologically derived wt viruses: APMV-2, -3, -4, -5, -7, and -9. Another virus was rAPMV-4, a recombinant derivative of wt APMV-4. The remaining three viruses, called rAPMV-2 (type 1 Africa), rAPMV-4/Fcs-BC, and rAPMV-7/Fcs-5B, were versions of wt rAPMV-2, -4, and -7, respectively, in which the naturally-occurring non-multi-basic F cleavage site was modified into a multi-basic site containing the optimal furin motif (Table 1). The animals were observed daily from days 0–10 and on days 12, 21 and 28 for any clinical signs of illness or distress. None of the animals exhibited any clinical signs of infection such as weight loss, increased body temperature, fever, or signs of respiratory distress, and no deaths were recorded. Thus, none of these APMV strains and cleavage site mutants was overtly pathogenic in rhesus macaques.

The article "Evaluation of the Replication, Pathogenicity, and Immunogenicity of Avian Paramyxovirus (APMV) Serotypes 2, 3, 4, 5, 7, and 9 in Rhesus Macaques" was retracted in 2020. Reasons: manipulated images; duplicated images; concerns about the data.

### Replication of APMV strains in the upper and lower respiratory tract of rhesus macaques

To evaluate replication of the APMVs in the upper respiratory tract of rhesus macaques, nasal washes were collected from days 0 to 10 and on days 12 and 21. Virus titers were determined by titration in embryonated chicken eggs, with the exception of APMV-5, which does not grow in chicken eggs. Thus, serial dilutions were prepared from the nasal washes and inoculated into the allantoic cavity of embryonated 9-day-old chicken eggs, and 4 dpi the allantoic fluid was collected and assayed for the presence of virus by HA assay. Virus titers were expressed as log_10_ EID_50_ per mL (Table 2). Replication of APMV-5 was determined by a limiting dilution assay on Vero cells in which virus-infected wells were detected by NA activity.

**Table 2:** Shedding of the indicated APMV strains from the upper respiratory tract of rhesus macaques.*

Virus	Animal No.	Nasal wash virus titer (log_10_ EID_50_) on indicated days †							
		0 1 2 3 4 5 6 7							
wt APMV-2	1	–	0.8	–	–	–	–	–	–
	2	–	0.8	–	–	–	1.8	–	–
	3	–	1.5	–	0.8	–	–	–	1.3
	4	–	1.5	–	–	–	1.5	–	–
	Mean ‡	–	1.1	0.4	0.5	0.4	1.0	0.4	0.6
rAPMV-2 (type1 Africa)	1	–	–	–	–	–	0.8	–	–
	2	–	–	–	–	–	–	–	–
	3	–	0.8	–	0.8	–	0.8	–	1.3
	4	–	1.5	1.5	2.5	1.5	0.8	1.3	–
	Mean	–	0.8	0.7	1.0	0.7	0.7	0.6	0.6
wt APMV-3	1	–	–	–	–	–	–	–	–
	2	–	–	–	1.4	2.3	1.8	–	1.3
	3	–	–	–	–	–	0.8	–	–
	4	–	0.8	–	–	–		–	–
	Mean	–	0.5	0.4	0.6	0.9	0.8	0.4	0.6
wt rAPMV-4	1	–	–	–	–	–	–	–	–
	2	–	–	–	–	–	–	–	–
	3	–	–	–	–	–	–	–	–
	4	–	–	–	–	–	–	–	–
	Mean	–	0.4	0.4	0.4	0.4	0.4	0.4	0.4
rAPMV-4/Fc-Bc	1	–	–	–	–	–	–	–	–
	2	–	–	–	–	–	–	–	–
	3	–	–	–	–	–	–	–	–
	4	–	–	–	–	–	–	–	–
	Mean	–	0.4	0.4	0.4	0.4	0.4	0.4	0.4
wt APMV-5 §	1	–	–	–	–	–	–	–	–
	2	–	–	–	–	–	–	–	–
	3	–	–	–	–	–	–	–	–
	4	–	–	–	–	–	–	–	–
	Mean	–	–	–	–	–	–	–	–
wt APMV-7	1	–	0.8	–	–	–	1.8	1.5	–
	2	–	1.5	–	–	2.3	2.3	0.8	–
	3	–	1.5	–	–	–	1.5	0.8	–
	4	–	0.8	–	0.8	0.8	–	–	–
	Mean	–	1.1	0.4	0.5	1.0	1.5	0.9	0.4
rAPMV-7/Fcs-5B	1	–	1.3	–	–	–	–	–	–
	2	–	0.8	–	–	–	–	–	–
	3	–	–	–	–	–	–	–	–
	4	–	–	–	–	–	–	–	–
	Mean	–	0.7	0.4	0.4	0.4	0.4	0.4	0.4
wt APMV-9	1	–	0.8	–	–	–	–	–	–
	2	–	1.3	–	–	–	–	–	–
	3	–	–	1.3	0.8	–	–	–	1.3
	4	–	1.3	1.5	1.5	2.6	1.3	1.3	–
	Mean	–	0.9	0.9	0.8	0.9	0.6	0.6	0.6

* Rhesus macaques in groups of four were inoculated simultaneously by the intranasal and intratracheal routes with a 1-ml inoculum per site containing 6.0 log_10_ PFU per ml of the indicated virus on day 0. Nasal washes were performed daily from day 0 to day 10 and on day 12.

† The 50 percent egg infectious dose (EID_50_) virus titer (expressed as log_10_ EID_50_ per mL), determined as described in Materials and Methods. Limit of detection was 0.8 log_10_ per mL. For calculation of daily means, a value of 0.4 was used for samples with no detectable virus.

‡ For calculation of daily means, a value of 0.4 log_10_ per mL was used for samples with no detectable virus.

§ Shedding of wt APMV-5 was measured by limiting dilution assay of nasal wash fluid on Vero cells, followed by virus detection using a neuraminidase assay.

The article "Evaluation of the Replication, Pathogenicity, and Immunogenicity of Avian Paramyxovirus (APMV) Serotypes 2, 3, 4, 5, 7, and 9 in Rhesus Macaques" was retracted in 2020. Reasons: manipulated images; duplicated images; concerns about the data.

Virus shedding from the upper respiratory tract was undetectable for 3 strains, namely wt rAPMV-4, rAPMV-4/Fc-BC, and wt APMV-5. For the other strains, low levels of shedding were detected in most of the animals. Specifically, wt APMV-2 was detected in nasal washes from all 4 animals on day 1, from 1 animal on day 3, 2 animals on day 5 and from 1 animal on day 7. The mean daily titers ranged from 0.8 to 1.1 log_10_ EID_50_ per mL, and the highest mean daily titer was detected on day 1. Replication of the recombinant version of APMV-2 with multi-basic F cleavage site derived from serotype 1 (Africa) was detected in 3 of 4 animals: 1 animal shed low titers of virus consecutively from days 1 to 6, another shed virus on 1 day, and another shed virus on 4 days. Shedding of wt APMV-3 was detected in 3 of 4 animals: 1 animal shed on days 3, 4, 5, and 7, while 2 animals shed detectable virus only on single days. Wt APMV-7 was isolated from all inoculated animals on day 1 and from either 1, 2 or 3 animals on days 3 to 6, whereas rAPMV-7/Fcs-5B was isolated only on day 1 from 2 animals and was not detected any of the animals on other days. Wt APMV-9 was detected on a single day (day 1) in 2 animals, while 2 animals shed over several days.

To evaluate the replication of APMVs in the lower respiratory tract of the inoculated animals, BALs were collected on days 2, 4, 6 and 8, and tracheal lavages were collected on days 10 and 12. All samples were processed and titrated as described above. Virus was detected only in the BAL samples (Table 3). Each strain except for wt APMV-5 replicated detectably in the lower respiratory tract of rhesus macaques. Specifically, wt APMV-2 was detected in all 4 animals on day 2, and in 1 or 2 animals on days 4 and 6, respectively (Table 3). Replication of rAPMV-2 (type 1 Africa) seemed to be more robust: virus shedding was detected from day 2 to day 6 in all of the animals, with mean daily titers ranging from 1.5 to 2.5 log_10_ EID_50_ per mL. Shedding of wt APMV-3 was detected in all inoculated animals until day 4, and in 2 animals until day 6, with mean daily titers of 0.9 to 2.2. Interestingly, while wt rAPMV-4 had not been detected in nasal washes from any animal, as described above (Table 2), this virus was detected on day 2 in BALs of 2 animals (Table 3). Similarly, the F cleavage mutant rAPMV-4/Fc-BC had not been detected in nasal wash specimens (Table 2), it was detected on days 2 and/or 4 in BALs of 3 of 4 inoculated animals. Whereas wt rAPMV-2 was detected in BALs only on day 2, the cleavage site mutant derivative was detected on days 2 and 4. Consistent shedding of wt APMV-7 and rAPMV-7/Fcs-5B was detected in all of the animals from days 2 to 6. Mean daily titers for the 2 viruses were similar and ranged from 1.2 to 3 log_10_ EID_50_ per mL. Thus, while it appeared that the cleavage site mutation Fcs-5B had a negative effect on replication of APMV7 in the upper respiratory tract (Table 2), it did not affect replication of APMV-7 in the lower respiratory tract (Table 3). Both versions of APMV-7 were detected more readily from the lower versus the upper respiratory tract. Wt APMV-9 was detected on day 2 in 3 of the 4 inoculated animals, and in 1 animal each on day 4 and 6.

The article "Evaluation of the Replication, Pathogenicity, and Immunogenicity of Avian Paramyxovirus (APMV) Serotypes 2, 3, 4, 5, 7, and 9 in Rhesus Macaques" was retracted in 2020. Reasons: manipulated images; duplicated images; concerns about the data.

**Table 3:** Detection of the indicated APMV strains from the lower respiratory tract of rhesus macaques.*

Virus	Animal No.	Virus titer in BAL (log_10_ EID_50_) on indicated days †				Sum of daily titers ‡
		2 4 6 8				
wt APMV-2	1	2.3	0.8	–	–	3.9
	2	1.5	–	1.8	–	4.1
	3	2.5	–	–	–	3.7
	4	2.3	1.5	–	–	4.6
	Mean §	2.1	0.8	0.7	0.4	4.1
rAPMV-2 (type1 Africa)	1	2.5	2.5	2.5	–	7.9
	2	2.5	1.5	1.8	–	6.2
	3	2.5	2.3	0.8	–	6.0
	4	2.5	1.5	0.8	–	5.2
	Mean	2.5	1.9	1.5	0.4	6.3
wt APMV-3	1	2.5	1.8	1.5	–	6.2
	2	1.5	1.5	–	–	3.8
	3	2.3	2.3	1.3	–	6.3
	4	2.5	1.5	–	–	4.8
	Mean	2.2	1.8	0.9	0.4	5.3
wt rAPMV-4	1	1.8	–	–	–	3.0
	2	0.8	–	–	–	2.0
	3	–	–	–	–	1.6
	4	–	–	–	–	1.6
	Mean	0.8	0.4	0.4	0.4	2.0
rAPMV-4/Fc-Bc	1	–	1.5	–	–	2.7
	2	–	–	–	–	1.6
	3	1.3	–	–	–	2.5
	4	1.5	0.8	–	–	3.1
	Mean	0.9	0.8	0.4	0.4	2.5
wt APMV-5 ¶	1	–	–	–	–	–
	2	–	–	–	–	–
	3	–	–	–	–	–
	4	–	–	–	–	–
	Mean	–	–	–	–	–
wt APMV-7	1	3.5	2.3	1.4	–	7.6
	2	2.8	1.5	1.5	–	6.2
	3	2.8	1.5	1.3	–	6.0
	4	2.8	1.8	0.8	–	5.8
	Mean	3.0	1.8	1.2	0.4	6.4
rAPMV-7/Fcs-5B	1	3.5	1.8	2.3	–	8.0
	2	2.5	3.5	0.8	–	7.2
	3	3.5	1.8	2.5	–	8.2
	4	2.5	1.5	0.8	–	5.2
	Mean	3.0	2.1	1.6	0.4	7.1
wt APMV-9	1	–	1.3	–	–	2.5
	2	2.3	–	–	–	3.5
	3	1.5	–	–	–	2.7
	4	0.8	–	0.8	–	2.4
	Mean	1.2	0.6	0.5	0.4	2.8

* This is a continuation of the experiment described in Table? 2. BAL was performed on days 2, 4, 6, and 8.

† The 50 percent egg infectious dose (EID_50_) virus titer (expressed as log_10_ EID_50_ per mL) was determined as described in materials and methods. Limit of detection was 0.8 log_10_ per mL.

‡ The sum of daily titers (area under the curve) was used to determine magnitude of virus shedding. A value of 0.4 was used for samples with no detectable virus.

§ For calculation of daily means, a value of 0.4 log_10_ per mL was used for samples with no detectable virus.

¶ Shedding of wt APMV-5 was determined by limiting dilution assay of BAL fluid on Vero cells, followed by virus detection using a neuraminidase assay.

The article "Evaluation of the Replication, Pathogenicity, and Immunogenicity of Avian Paramyxovirus (APMV) Serotypes 2, 3, 4, 5, 7, and 9 in Rhesus Macaques" was retracted in 2020. Reasons: manipulated images; duplicated images; concerns about the data.

For an overall comparison of virus replication in the lower respiratory tract, the sum of the daily BAL titers from days 2 to 8 was calculated for each animal, and the mean sum of daily titers of each virus was calculated (Table 3). This identified wt rAPMV-4, rAPMV-4/Fc-BC, and wt AMPV-9 as the viruses with the lowest level of replication in the lower respiratory tract [in the order: wt rAPMV-4 (2.0 log_10_) < rAPMV/4Fc-BC (2.5 log_10_) < wt APMV-9 (2.8 log_10_)]. Wt APMV-2 and wt APMV-3 replicated to slightly higher overall levels [wt APMV-2 (4.1 log_10_) < wt APMV3 (5.3 log_10_)], while rAPMV-2 (type 1 Africa), wt APMV-7, and rAPMV7/Fcs-5B were identified as the viruses with the highest mean sum of daily titers [rAPMV-2 (type 1 Africa) (6.3 log_10_) < wt APMV-7 (6.4 log_10_) < rAPMV7/Fcs-5B (7.1 log_10_)]. Interestingly, the mean sum of daily titers of rAPVM-2 with F cleavage site from type 1 Africa was significantly higher than that of wt rAPMV2, showing that the replacement of the F cleavage site by that of type 1 Africa significantly increased the replication of APMV-2 in the lower respiratory tract (One Way Anova with Tukey post-hoc analysis).

In summary, APMV of serotypes 2, 3, 7 and 9, and derivatives thereof with F cleavage site mutations replicated in rhesus macaques at a low-to-moderate level over a period of days. rAPMV-2 (type 1 Africa) and wt APMV7 showed the most consistent replication in both the upper and lower respiratory tract of rhesus macaques. Replication of APMV serotype 4 was undetectable in the upper respiratory tract; in the lower respiratory tract, a low level of shedding, close to the level of detection, was detected. No virus shedding was detectable from the upper or lower respiratory tract for any of the viruses after day 7 post-infection, indicating that replication of all of these viruses was self-limiting. Furthermore, there was no detectable spread of the any of these APMVs to the gastrointestinal tract (not shown). Only one of the viruses tested, namely wt APMV-5, could not be detected nasal washes or BAL from any of the inoculated animals.

### APMV serotype-specific serum antibody responses

Serum samples of the rhesus macaques infected with the various APMV strains were collected on days 0, 21 and 28 dpi. Serotype-specific serum antibody titers were determined by a modified HI assay using chicken erythrocytes, except in the case of APMV-5, in which case titers were determined by an NI assay in Vero cells (Table 4). All the animals were confirmed to be seronegative for APMV-specific antibodies on day 0. Each of APMV serotypes induced a serum antibody response. However, the magnitude of the response varied. On day 21, the highest mean HI antibody titers were observed in rhesus macaques immunized wt APMV-2 (7.00 log_2_ ± 1.4). Moderate mean HI antibody titers were observed with wt APMV-3 (5.8±0.5), wt APMV-7 (5.3±0.5), rAPMV-7/Fcs-5B (4.5±0.6) and wt APMV-9 (4.50±0.6), and the lowest mean HI antibody titers were observed with rAPMV-2 (type 1 Africa) (3.3±0.5) and wt APMV-5 (2.5±1.7). In case of wt rAPMV-4 and rAPMV-4/Fc-BC, only two of the four animals had serum HI antibody responses. The mean HI antibody titer values determined on day 28 were similar to day 21 values.

The article "Evaluation of the Replication, Pathogenicity, and Immunogenicity of Avian Paramyxovirus (APMV) Serotypes 2, 3, 4, 5, 7, and 9 in Rhesus Macaques" was retracted in 2020. Reasons: manipulated images; duplicated images; concerns about the data.

**Table 4:** Serum antibody responses in rhesus macaques infected with the indicated APMV.*

Virus	Animal No.	HI antibody titer † (mean reciprocal log_2_ ± standard error)		Neutralizing antibody titer ‡ (mean reciprocal log_2_ ± standard error
		Day		Day
		21	28	28
wt APMV-2	1	7	7	2
	2	8	7	3
	3	5	5	2
	4	8	7	5
	Mean	7.0±1.4	6.5±1.0	3.0±1.4
rAPMV-2 (type1 Africa)	1	3	3	0
	2	3	3	0
	3	3	3	0
	4	4	4	0
	Mean	3.3±0.5	3.3±0.5	0
wt APMV-3	1	6	6	7
	2	6	6	7
	3	6	6	5
	4	5	5	6
	Mean	5.8±0.5	5.8±0.5	6.3±1.0
wt rAPMV-4	1	3	4	7
	2	0	0	6
	3	0	0	5
	4	4	4	6
	Mean	1.8±2.1	2.0±2.3	6.0±0.8
rAPMV-4/Fc-Bc	1	0	0	4
	2	4	4	6
	3	0	0	4
	4	3	3	5
	Mean	1.8±2.1	1.8±2.1	4.8±1.0
wt APMV-5 §	1	3	3	3
	2	3	3	3
	3	0	0	0
	4	4	4	0
	Mean	2.5±1.7	2.5±1.7	1.5±1.7
wt APMV-7	1	5	5	3
	2	5	5	3
	3	6	7	6
	4	5	6	5
	Mean	5.3±0.5	5.8±1.0	4.3±1.5
rAPMV-7/Fcs-5B	1	4	4	2
	2	5	5	4
	3	5	5	3
	4	4	4	2
	Mean	4.5±0.6	4.5±0.6	2.8±1.0
wt APMV-9	1	5	6	10
	2	5	5	9
	3	4	4	9
	4	4	5	10
	Mean	4.5±0.6	5.0±0.8	9.5±0.6

* This is continuation of the experiment described in Tables? 2 and 3. Serum samples were collected before inoculation on day 0, and after inoculation on days 21 and 28.

† The hemagglutination inhibition (HI) titer is expressed as the mean reciprocal log_2_ (± standard errors of the mean) of the highest serum dilution causing complete inhibition of four HA units of the indicated APMV, except for APMV-5, which was evaluated by neuraminidase inhibition (NI) assay. All the values are averages from three independent experiments. The mean serum HI titers in all the day 0 serum samples were 0.

‡ The serum neutralizing antibody titers were expressed as mean reciprocal log_2_ of the serum dilution resulting in complete neutralization of infection in 50% of the wells (mean ± standard errors of the mean). The limit of detection is 0. The mean neutralizing antibody titers in all the day 0 serum samples were 0.

§ The antibody response to APMV-5 was evaluated by NI assay as described in Materials and Methods. The NI titer is expressed as the mean reciprocal log_2_ (± standard errors of the mean) of the highest serum dilution causing neuraminidase inhibition.

The article "Evaluation of the Replication, Pathogenicity, and Immunogenicity of Avian Paramyxovirus (APMV) Serotypes 2, 3, 4, 5, 7, and 9 in Rhesus Macaques" was retracted in 2020. Reasons: manipulated images; duplicated images; concerns about the data.

The ability of the serum samples collected on day 28 to neutralize the respective APMV serotype was assessed by a micro-neutralization assay (Table 4). The antisera from the monkeys immunized with wt APMV-9 had the highest mean neutralizing antibody titer of log_2_ 9.5±0.6. The next highest titer was observed in monkeys infected with wt rAPMV-3 (6.3±1.0). The neutralizing antibody titer in monkeys infected with other serotypes decreased in the order: wt rAPMV-4 (6.0±0.8) > rAPMV-4/Fc-BC (4.8±1.0) > wt APMV-7 (4.3±1.5) > wt APMV-2 (3.0±1.4) > rAPMV-7/Fcs-5B (2.8±1.0). Surprisingly, serum neutralizing antibodies were not detected in the case of rAPMV-2 (type 1 Africa). In this study, no direct correlation was found between HI titer and neutralizing titer.

In addition, we examined the serum samples collected on day 28 from rhesus monkeys for reactivity against different APMV proteins in purified virions from egg allantoic fluids by Western blotting assay (Fig. 1). We did not examine APMV-5 because infectious virus was not recovered from any of the animals, and thus infectivity is minimal or negative. We probed the Western blots with pre-immune and immune serum samples from all the four monkeys infected with each of the other APMVs. Every animal reacted to the respective NP, F_1_, P and M proteins with varying degrees of intensities when 5 µg of each APMV virus preparation were run on the gels and blotted to nitrocellulose. For the HN and F_0_ proteins, reactive bands were recognized to varying extents or not at all by sera from individual animals, which is consistent with the known drastic changes in immune reactivity of paramyxovirus HN and F proteins when denatured [50]. All pre-immune serum samples were found negative.

**Figure 1:** Analysis of the reactivity of sera from rhesus macaques collected following infection with the indicated APMVs, evaluated by Western blotting against purified virus of the homologous APMV strain. Virus representing each of the indicated APMV strains was purified from sucrose gradient centrifugation from allantoic fluid from infected eggs, and was denatured and reduced and subjected to 10% SDS-PAGE under reducing conditions and transferred to nitrocellulose membranes. The membranes were cut into strips and incubated with 1∶500 dilutions of day 0 and 28 sera from each of the monkeys in each group. The positions of the HN, F_0_, NP, F_1_, P and M proteins are indicated. The positions and sizes (kDa) of size markers are indicated to the left.

The article "Evaluation of the Replication, Pathogenicity, and Immunogenicity of Avian Paramyxovirus (APMV) Serotypes 2, 3, 4, 5, 7, and 9 in Rhesus Macaques" was retracted in 2020. Reasons: manipulated images; duplicated images; concerns about the data.

## Discussion

APMVs are frequently isolated from wide variety of avian species around the world and have been grouped into nine established serotypes, although two additional serotypes have been provisionally identified (Introduction). Among the nine established serotypes, APMV-1 (NDV) is the most extensively characterized due to its importance as a major pathogen of poultry. APMV serotypes 2 to 9 are frequently isolated from both domestic and wild birds, but have been largely uncharacterized until recently. NDV has been shown to infect not only avian species but also non-avian species, although its replication is restricted in non-avian hosts [29], [30]. NDV is being developed as promising viral vaccine vector for delivery of a number of antigens of animal and human pathogens [51]. However, the potential of APMV-2 to -9 as vaccine vectors for humans was not known. Previously, we demonstrated the replication of APMV-2 to -9 in hamsters and mice [4], [5]. However, low phylogenetic and anatomic relatedness between the rodent models and humans necessitate the use of more relevant models for assessment of replication and pathogenicity of APMV-2 to -9.

Therefore, the goal of this study was to evaluate the replication and pathogenicity of a number of non-NDV APMV serotypes in non-human primates. Rhesus macaques were evaluated for permissiveness to infection, clinical disease, magnitude of replication, shedding and induction of antibodies. Rhesus macaques have been used commonly as a non-human primate model to study replication and pathogenicity of various viruses, to screen attenuation phenotypes of live virus vaccines, and to evaluate immune responses of virus vaccine candidates. The safety, immunogenicity, and protective efficacy of NDV has also been demonstrated in this model [29]–[33], [51].

In this study, we chose to evaluate nine different APMV strains. Six of these were wt viruses representing six different serotypes, specifically biologically-derived wt APMV -2, -3, -5, -7, and -9, as well as a recombinant version of wt APMV-4. We chose wt APMV-2, -5, -7 and wt rAPMV-4 because we previously showed that replication of these viruses in cell culture does not require, and is not enhanced by, exogenous protease supplementation [8], [11], [13], [19]. Since this property is known to correlate with pantropic replication and virulence by NDV in chickens, it was possible that it might confer increased replication of these non-NDV APMVs in the rhesus macaques, although we note that this NDV paradigm had not been consistent for these non-NDV APMVs in chickens [16], [18], [19]. Wt APMV-3 was selected because this virus replicates to high titer in cell culture and a reverse genetics system has been developed for this serotype [9], [17]. Wt APMV-9 was selected because this virus replicates well in nasal turbinate and lungs of mice and hamsters [4], [5]. The other three viruses evaluated in this study were recombinant versions of APMV-2, -4, and -7 in which the naturally-occurring F protein cleavage sites were replaced by multi-basic cleavage sites containing the optimal furin motif. Specifically, rAPMV-2 (type 1 Africa) contained the multi-basic cleavage site RRRRR↓F that is present in a virulent African NDV strain; rAPMV-4/Fc-BC contained the cleavage site RRQKR↓F derived from the mesogenic NDV strain Baudette C; and rAPMV-7/Fcs-5B contained the cleavage site RRKKR↓F derived from the velogenic NDV strain Nigeria/95. As noted, in NDV, multi-basic cleavage sites generally are associated with greater virulence in chickens.

The article "Evaluation of the Replication, Pathogenicity, and Immunogenicity of Avian Paramyxovirus (APMV) Serotypes 2, 3, 4, 5, 7, and 9 in Rhesus Macaques" was retracted in 2020. Reasons: manipulated images; duplicated images; concerns about the data.

Rhesus macaques infected with APMV-2, -3, -4, -5, -7 and -9 showed no signs of any disease. APMV-2, -3, -7, and -9 replicated to low titers in upper respiratory tract as evidenced by low level of shedding of these viruses in nasal washes of animals from day 1 to 7. APMV-4 and -5 were found negative for shedding from upper respiratory tract. Similarly, we previously showed that rhesus macaques or African green monkeys that were infected by the combined intranasal and intratracheal routes with NDV strain BC were mostly negative for viral shedding [29]. Together, these results indicate that APMVs are highly restricted in replication in the upper respiratory tract of monkeys. However, analysis of BAL samples in the present study revealed replication of all these APMVs except wt APMV-5 in lower respiratory tract until day 6 post infection, although at different levels. The magnitude of shedding of wt APMV-2, rAPMV-2 (type 1 Africa), wt APMV-3, wt APMV-7, and rAPMV-7/Fcs-5B was moderate, while in case of wt APMV-9, wt rAPMV-4, and rAPMV-4/Fc-BC it was low. In contrast, a very low level of shedding (as determined by plaque assay of tracheal lavages or samples of lung tissues) was detected from lower respiratory tract of AGMs infected with NDV in earlier studies [29]. This indicates that, compared to NDV, wt and recombinant APMV-2 and 7, and wt APMV-3 replicate more efficiently in the lower respiratory tract in non-human primates. This apparent increased replication may provide an advantageous increase in immunogenicity for an expressed foreign antigen. Despite the somewhat greater replication of certain APMVs in the respiratory tract, analysis of fecal samples of rhesus macaques infected with all these APMVs revealed no shedding, suggesting a lack of spread to the gastrointestinal tract. These observations suggest that like NDV, APMV-2, -3, -4,-7 and -9 are highly restricted and highly attenuated in non-human primates.

The article "Evaluation of the Replication, Pathogenicity, and Immunogenicity of Avian Paramyxovirus (APMV) Serotypes 2, 3, 4, 5, 7, and 9 in Rhesus Macaques" was retracted in 2020. Reasons: manipulated images; duplicated images; concerns about the data.

For a number of the APMV strains, replication in the upper respiratory tract appeared to be less efficient compared to the lower respiratory tract. One possible explanation is that there might be a lower density of APMV receptors in the upper respiratory tract of non-human primates compared to lower respiratory tract, and hence a lower level of replication. A second possible factor is that birds have a higher body temperature compared to primates. Therefore, both the upper and lower respiratory tract of primates may be suboptimal for APMV replication, and this effect would be more pronounced in the upper respiratory tract due to its relatively lower temperature. The low level of shedding of APMVs from upper respiratory tract of non-human primates predicts that shedding also should be reduced from humans, which would limit release into the environment and would be a desirable feature for a vaccine vector.

We previously showed that, whereas wt APMV-2, -4, and -7 did not form syncytia or plaques in cell culture, despite their independence from added protease, in each case the introduction of the respective multi-basic site resulted in a gain-in-function conferring the ability to form syncytia and plaques [16], [18], [19]. The introduction of the multi-basic sites also increased virus replication in vitro - by 10-fold [16], [18], [19]in the case of rAPMV-2 (type 1 Africa) and rAPMV-7/Fcs-5B, and by 500- to 5000-fold in the case of rAPMV-4/Fc-BC. However, there was no observed difference in replication or pathogenicity in chickens [16], [18], [19]. For the purpose of developing APMV vaccine vectors for possible human use, these mutations had at least two potential advantages. First, the increased growth in vitro would facilitate vaccine manufacture. Second, the cleavage site mutations might increase vector replication in primates, in which case a modest increase in replication might increase the immunogenicity of an expressed foreign antigen while retaining the attenuation phenotype. In the present study, the introduction of the multi-basic sites were associated with an apparent increase in replication in the case of rAPMV-2 (type 1 Africa), and possibly a marginal increase in the case of rAPMV-4/Fc-BC, and an apparent decrease in replication in the case of rAPMV-7/Fcs-5B. With respect to the absence of clinical disease, the mutants remained as attenuated as their wt parents. However, a larger study would be required to confirm these preliminary observations.

The article "Evaluation of the Replication, Pathogenicity, and Immunogenicity of Avian Paramyxovirus (APMV) Serotypes 2, 3, 4, 5, 7, and 9 in Rhesus Macaques" was retracted in 2020. Reasons: manipulated images; duplicated images; concerns about the data.

A single inoculation via combined intranasal and intratracheal routes in rhesus macaques with wt APMV-2, wt APMV-3, wt APMV-7, rAPMV-7/Fcs-5B and wt APMV-9 induced substantial HI antibody titer, whereas serum HI antibody responses induced by rAPMV-2 (type 1 Africa), wt rAPMV-4, rAPMV-4/Fc-BC, and wt APMV-5 was low. The HI titers correlated either completely or partially with the level of shedding from the lower respiratory tract except in the case of wt APMV-5, for which no shedding was observed but a low level of NI titer was produced. To date, APMV-5 has only been isolated from budgerigars, which are thought to be its natural host [24]. These observations indicated that this virus probably is strongly host restricted.

In this study, no direct correlation was found between HI titer and neutralization titer. In the cases of wt APMV-3, rAPMV-4, rAPMV-4/Fc-BC, and wt APMV-9, the neutralization titers were higher compared to the HI titers, whereas the converse was true for the remaining APMVs. Since HI titers reflect antibodies specific for the attachment site of HN whereas neutralizing antibodies reflect broader antibody responses against antigenic sites throughout the HN and F proteins, the instances of relatively higher neutralizing titers might reflect a disproportionately greater contribution from additional epitopes in the HN and F proteins.

The serum HI antibody titers induced in rhesus monkeys by wt APMV-2, wt APMV-3, wt APMV-7, rAPMV-7/Fcs-5B, and wt APMV-9 was either higher or equal to the HI antibody titers induced by mesogenic NDV strain BC in African green monkeys in previous studies [52]. These serotypes are thus candidates for further development as vaccines for human use. In the cases of wt rAPMV-4, rAPMV-4/Fc-BC, and wt APMV-5 (where not all of the monkeys seroconverted) and rAPMV-2 (type 1 Africa), the HI antibody titers were lower than that induced by NDV in a previous study [52], suggesting that these serotypes are less promising. One incongruity in the present study is the low titers of HI antibodies, and lack of detectable neutralizing antibodies, induced by rAPMV-2 (type 1 Africa) despite the relatively robust replication of this vector and compared to the greater immunogenicity of its wt APMV-2 parent despite the lower replication of the parent.

In summary, we have evaluated the replication and pathogenicity of APMV serotypes-2, -3, -4, -5, -7, and -9 in non-human primates. These respiratory viruses are highly restricted for replication in respiratory tract of rhesus macaques. We have also demonstrated a substantial level of immunogenicity for wt APMV-2, -3 -7 and -9 and recombinant wt APMV-4, APMV-4/Fc-BC, and APMV-7/Fcs-5B in this non-human primate model. As these APMVs are serologically distinct from NDV and from each other, they may be developed as vectors and used in heterologous prime-boost combinations to induce robust systemic and mucosal immune responses against foreign antigens.
